# Identification of Novel CircRNA-miRNA-mRNA Regulatory Network and Its Prognostic Prediction in Breast Cancer

**DOI:** 10.1155/2021/2916398

**Published:** 2021-10-29

**Authors:** Rui Huang, Hao Yu, Xiao Zhong

**Affiliations:** ^1^Department of Oncology, People's Hospital of Jiangxi Province, Nanchang, China; ^2^Organization Department, Jiangxi Health Vocational College, Nanchang, China; ^3^Clinical Psychology, Jiangxi Corning Hospital, Nanchang, China

## Abstract

**Aim:**

This study aimed to investigate the expression profiles of circRNAs and candidate circRNA-miRNA-mRNA network in BC.

**Methods:**

Differentially expressed circRNAs, miRNAs, and mRNAs (DEcircRNAs, DEmiRNAs, and DEmRNAs) between BC and normal breast tissue samples were screened by analyzing raw data of the RNA sequencing profile. The expression levels of hub genes in 48 pairs of cancerous and tumor-free breast tissues surgically resected from BC patients were determined by RT-qPCR analysis.

**Results:**

A total of 145 DEcircRNAs, 140 DEmiRNAs, and 2451 DEmRNAs between BC and normal breast tissue samples were screened out. There were 5 pairs of upcircRNA-downmiRNA-upmRNA network and 20 pairs of downcircRNA-upmiRNA-downmRNA network. EIF4EBP1, DUSP1, EGR2, EZH1, and CBX7 were found to be correlated with overall survival of the patients with BC. The expression level of EIF4EBP1 was increased and the expression levels of DUSP1, EGR2, EZH1, and CBX7 were decreased in cancerous breast tissues compared to tumor-free breast tissues (*p* < 0.0001). The RT-qPCR results from 48 BC patients were consistent with the bioinformatics results.

**Conclusion:**

This study provides a novel perspective to study circRNA-miRNA-mRNA network in BC and assists in the identification of new potential biomarkers to be used for diagnostic and prognostic purposes.

## 1. Introduction

Breast tissue consists of 15 to 20 lobules, which is connected to nipples, connective tissue, adipose tissue, and lymphoid tissue through mammary ducts. Breast cancer (BC) is commonly seen in lobules [1]. No common symptoms are involved in BC except for painless breast lump in the breast. In the early stage of the disease, BC may be characterized by axillary lymphadenopathy. However, some symptoms, which are rarely seen, such as hemorrhagic nipple discharge, redness, and breast deformity or invagination, are the risk factors of malignant tumor of breast [2]. BC is the most common form of cancer among females. It is the second-leading cause of cancer deaths which closely followed lung cancer. For years, BC has been one of the top ranked cancers in females, regardless of incidence rate or mortality rate. It is estimated that 2.1 million people were diagnosed with BC worldwide in 2020, and 9.6 million of global population out of 18.1 million (new cancer cases) died due to cancer, of which BC deaths accounted for about 11.6% [3]. Most BCs are permeable, which have spread from ducts and glands to surrounding tissues and lymph nodes. At present, there are 4 main subtypes of BC, including luminal A, luminal B, HER2-overexpression, and basal-like, which behave differently in terms of onset age and prognosis [4]. Females are more likely to suffer from BC, and the incidence cases in females are 100 times higher than that in males [5].

BC is a metastatic tumor, which can spread to distant organs such as bone, liver, lung and brain, resulting in low cure rate. Early diagnosis, such as mammography and magnetic resonance imaging, helps to improve prognosis and survival [6, 7]. Genetic and non-genetic factors, such as gender, age, estrogen, and unhealthy lifestyle, have been identified as the risks of BC. In most cases, there is no clear inheritance pattern [8]. Numerous studies demonstrated that the increase of individual risk in BC was associated with genes, and it was estimated that the proportion of familial aggregation genetic factors and environmental factors in BC was 73% and 27%, respectively. In addition, genetic factors also lead to a lower age of onset [9]. In general, the etiology of BC is supposed to be associated with three types of genes, including high-risk genes such as BRCA1 and BRCA2 [10], moderate-risk genes such as CHEK2, ATM, and PALB2 [11], and low-risk genes such as SNPs [12]. Circular RNAs (circRNAs), as one of endogenous non-coding RNAs (ncRNAs), are more abundant than messenger RNA (mRNA), which is expressed in highly divergent eukaryotes [13]. In recent years, the regulation role of circRNA in human cancers, such as lung cancer [14], liver cancer [15], gastric cancer [16], and BC [17], has been revealed in many studies. In addition, more studies on the potential function of circRNA as a microRNA (miRNA) sponge or RNA protein complexes regulating gene transcription in cancer have been confirmed, such as a novel circRNA named circIRAK3 in BC [18] and circMTO1 in hepatocellular carcinoma [19].

Although great progress has been made on the genetic factors related to BC pathogenesis, the function and clinical significance of some identified risk genes are limited due to lack of reliable risk estimation and unclear polygenic background. In this study, the synergism of the gene regulatory network of circRNA-miRNA-mRNA on the pathogenesis of BC was mainly analyzed, which contributed to a depth of understanding in various biological processes of BC and provided new potential biomarkers for diagnosis and prognosis.

## 2. Methods

### 2.1. Acquisition of Expression Profiles and Differential Analysis

The RNA sequencing profile of BC patients was obtained from the Cancer Genome Atlas (TCGA, https://tcga-data.nci.nih.gov/) database, including 1104 BC and 113 normal breast tissue samples.

Gene Expression Omnibus (GEO, https://www.ncbi.nlm.nih.gov/gds) stored a microarray dataset (accession numbers: GSE101123, submission date: Jul 11, 2017; last update date: Jul 25, 2021). 8 BC and 3 normal breast tissue samples were contained in the microarray dataset. Differentially expressed circRNAs, miRNAs, and mRNAs (DEcircRNAs, DEmiRNAs, and DEmRNAs) between BC and normal breast tissue samples were screened by analyzing raw data of the RNA sequencing profile and GSE101123 using the Limma package from the R/Bioconductor software in accordance with |log_2_ (fold change [FC])| > 1 and adjusted *p* ≤ 0.05.

### 2.2. CircRNA-miRNA-mRNA Regulatory Network Construction

(1) starBase database (https://starbase.sysu.edu.cn/index.php) was applied to perform a computer-based prediction of DEcircRNA-miRNA pairs; (2) MiRanda (https://www.cs.kent.ac.uk/people/staff/dat/miranda/), miRDB (http://mirdb.org/), miTarBase (https://miRTarBase.cuhk.edu.cn/), miRMap (https://mirmap.ezlab.org/), and TargetScan (http://www.targetscan.org/vert_71/) were considered as five miRNA-mRNA target prediction databases, which mapped DEmRNAs for miRNA-DEmRNA pairs of interest; (3) DEmiRNAs and common miRNAs among DEcircRNA-miRNA pairs and miRNA-DEmRNA pairs were overlapped for final circRNA-miRNA-mRNA regulatory network based on the principle of ceRNA network. The circRNA-miRNA-mRNA ceRNA network was constructed and visualized by using Cytoscape 3.4.0 software.

### 2.3. Functional Annotation for Genes of Interest

GO terms, as a global standard classification system, are used to describe the enrichment of biological function of gene. GO functional annotation covers biological process (BP), cellular component (CC), and molecular function (MF). Different genes coordinate with each other to perform biological functions. The pathways, including fundamental biochemical metabolism and signal transduction related to target genes, are determined by *p* value ≤ 0.05 as cutoff value using “clusterProfiler” package in R/Bioconductor. KEGG, known as public system database, is used to systematically analyze gene networks and molecular networks. Most known metabolic pathways and some known regulatory pathways are included in graphical maps of biochemical pathways, which are displayed in the KEGG pathway database. The Fisher test according to hypergeometric distribution is carried out to KEGG enrichment analysis using “clusterProfiler” package in R/Bioconductor, and finally the significance level (*p* value) of each pathway is calculated. *p* value ≤ 0.05 indicates that the screening criteria are significant.

### 2.4. Screening of Hub Genes by PPI Network

Search Tool for the Retrieval of Interacting Genes (STRING online tool, https://string-db.org) was applied to screen the DEGs. If the interactions with a medium confidence >0.4, it means that the interaction of hub genes is significant. The Cytoscape plugin cytoHubba was employed to construct the integrated regulatory networks.

### 2.5. Prediction and Evaluation of Prognosis-Related Hub Genes for BC

We collected the data, which were downloaded from TCGA database, of clinical samples and expression profiles of BC patients, so as to analyze the correlation between hub genes and overall survival of BC patients. According to hub gene expression, data of patient survival were collected by a receiver operating characteristic (ROC) curve.

### 2.6. Clinical Sample Collection

We collected 48 pairs of cancerous and tumor-free breast tissues surgically resected from BC patients who were admitted to Jiangxi Provincial People's Hospital from January 2020 to January 2021. No patients had received radiotherapy or chemotherapy before tissue specimen collection. Human tissue specimens were included using informed consent for a protocol approved by the Ethics Committee of Jiangxi Provincial People's Hospital.

### 2.7. Real-Time Quantitative Polymerase Chain Reaction (RT-qPCR) Validation

Firstly, TRIzol reagent (Invitrogen, Carlsbad, CA, USA) was used to extract total RNA from cancerous and tumor-free breast tissues and then the PrimeScript RT kit (Takara, Dalian, China) was applied for generation of cDNA. Finally, RT-qPCR through a StepOnePlus Real-Time PCR system (Applied Biosystems, Foster City, CA, USA) was performed using a SYBR-Green PCR kit (Roche Diagnostics, Indianapolis, IN, USA).  Table 1 lists the sequence information of the primers used for the qPCR. The results were analyzed using the 2-ΔΔ*Ct* method.

## 3. Results

### 3.1. Identification of DEcircRNAs, DEmiRNAs, and DEmRNAs in BC

We differentially analyzed the RNA sequencing profile of BC patients downloaded from TCGA database, including 1104 BC and 113 normal breast tissue samples, and screened out 140 DEmiRNAs (59 upregulated miRNAs and 81 downregulated ones) (Figure 1) and 2451 DEmRNAs (1231 upregulated mRNAs and 1220 downregulated ones). Furthermore, we differentially analyzed raw microarray data of the GSE101123 and found that 145 circRNAs were differentially expressed between 8 BC and 3 normal breast tissue samples, including 82 upregulated circRNAs and 63 downregulated ones (Figure 1).

### 3.2. GO Enrichment and KEGG Pathway Analysis of DEmRNAs in BC

Next, we performed functional enrichment analysis of GO and KEGG to study the biological function of DEmRNAs in BC.  Figure 2(a) shows top 15 GO biological processes significantly enriched (all *p* < 0.05) by DEmRNAs based on BP, CC, and MF categories. The enrichment results related to BP category revealed that the regulation of cell migration (GO: 0030334), anatomical structure morphogenesis (GO: 0009653), and regulation of cell motility (GO: 2000145) were abundant in DEmRNAs. Considering the enrichment results of the CC category, DEmRNAs were mainly enriched in collagen-containing extracellular matrix (GO: 0062023), contractile fiber (GO: 0043292), and sarcomere (GO: 0030017). With regard to the enrichment results of the MF category, DEmRNAs were mostly enriched in actin binding (GO: 0003779), calcium ion binding (GO: 0005509), and heparin binding (GO: 0008201).  Figure 2(b) shows top 15 KEGG pathways significantly enriched (all *p* < 0.05) by DEmRNAs. It was revealed that the DEmRNAs between BC and normal breast tissues were significantly enriched in focal adhesion (hsa04510), PPAR signaling pathway (hsa03320), ECM-receptor interaction (hsa04512), PI3K-Akt signaling pathway (hsa04151), axon guidance (hsa04360), and pathways in cancer (hsa05200).

### 3.3. Construction of CircRNA-miRNA-mRNA Regulatory Network in BC

In order to establish the circRNA-miRNA-mRNA ceRNA regulatory network, we firstly search the starBase database for miRNAs targeted by DEcircRNAs, miRanda, miRDB, miRMap, miTarBase, and TargetScan databases for DEmRNA-targeted miRNAs, with overlapped miRNAs obtained. DEmiRNAs and the overlapped miRNAs were intersected for construction of final circRNA-miRNA-mRNA regulatory network. According to ceRNA hypothesis that transcripts, including circRNAs, share microRNA (miRNA) binding sites and compete for post-transcriptional control, there are two paradigms of ncRNA regulation including upcircRNA-downmiRNA-upmRNA network and downcircRNA-upmiRNA-downmRNA network. There were 26 pairs of upcircRNA-downmiRNA-upmRNA network (Figure 3(a)) and 85 pairs of downcircRNA-upmiRNA-downmRNA network (Figure 3(b)).

### 3.4. Key CircRNA-miRNA-mRNA in Subnetwork

PPI network was constructed based on the DEmRNAs between BC and normal breast tissue samples mapped into the STRING database. 14 nodes, including 12 downregulated DEGs and 2 upregulated DEGs, and 9 interactions existed in the PPI network (Figure 4).

HMGA1 and EIF4EBP1 were upregulated hub genes, and DUSP1, JUN, EGR2, KAT2B, PER2, CRY2, TEF, WASF3, KDR, RRAGD, EZH1, and CBX7 were downregulated hub genes in BC. Based on the above hub genes in BC, the circRNA-miRNA-mRNA network was reconstructed. As shown in Figures 5(a) and 5(b) and Table 2, there were 5 pairs of upcircRNA-downmiRNA-upmRNA network and 20 pairs of downcircRNA-upmiRNA-downmRNA network.

### 3.5. Prognostic Value of Hub-Gene Signature in BC

The relationship between hub genes and overall survival of BC was analyzed by Kaplan–Meier and log-rank tests using expression profiles of breast invasive carcinoma samples in TCGA database. A total of 5 hub genes, EIF4EBP1, DUSP1, EGR2, EZH1, and CBX7, were found to be correlated with overall survival of the patients with BC (Figure 6). In addition, expression patterns of 5 hub genes were also investigated using the starBase database, and we found that EIF4EBP1 was displayed in high expression level in BC samples, whereas DUSP1, EGR2, EZH1, and CBX7 were exhibited in low expression level in BC samples (Figure 7).

### 3.6. RT-qPCR Validation

To check the credibility of the bioinformatics results, we determine the expression levels of EIF4EBP1, DUSP1, EGR2, EZH1, and CBX7 in the cancerous and tumor-free breast tissues by RT-qPCR analysis. Results were expressed as mean ± standard deviation and analyzed by using paired *t*-test. The expression level of EIF4EBP1 was increased, and the expression levels of DUSP1, EGR2, EZH1, and CBX7 were decreased in cancerous breast tissues compared to tumor-free breast tissues (*p* < 0.0001, Figure 8). The RT-qPCR results from 48 BC patients were consistent with the bioinformatics results.

## 4. Discussion

BC is found as one of major health public issues, which ranks the second cause of cancer-associated death among various females. BC is a heterogeneous group of diseases with variable morphologic and biological features [20]. Approximately 70–75% of BC is associated with positive hormone receptor [21]. Anti-hormone therapy is the standard treatment for majority of BC. However, 25–30% of BC females are at risk of recurrence due to endocrine resistance [22]. Therefore, it is of great clinical significance to find new biomarkers and clarify the pathogenesis of BC. CircRNA, some of which are considered as prognosis and diagnosis biomarkers, has been involved in tumor progression having a crucial role [23, 24]. However, previous studies of BC had limitations in differential expression of circRNAs, such as focus on one or several expressions. The potential circRNA network in BC has been rarely reported. LncRNAs associated with potential superior biomarkers of BC, as well as the interaction among circRNA, miRNAs, and mRNAs on the basis of circRNA network construction, were mainly explored in this study. According to TCGA and GSE101123 database analysis of breast tissue samples in BC and healthy people, differential expressions in the BC-specific circRNAs, miRNAs, and mRNAs were identified.

The interaction of gene expression was analyzed by GO term and KEGG pathways. GO term outcomes indicated that mRNAs were enrichment in some functions including cellular functions, immune functions, and metabolism functions. The results of KEGG pathway analysis showed that the specific mRNAs were highly associated with focal adhesion, PPAR signaling pathway, ECM-receptor interaction, PI3K-Akt signaling pathway, axon guidance, and other pathways in BC. Focal adhesion, as a non-receptor tyrosine kinase, has an important role in regulating cell migration, invasion, adhesion, proliferation, and survival in ovarian cancer [25]. The previous study supported that PI3K-Akt signaling pathway was associated with reduced apoptosis, cell growth stimulation, and increased cell proliferation [26]. PPAR signaling pathway is involved in the regulations of lipid metabolism, lipogenesis, maintenance of metabolic homeostasis, and expression of inflammation-related genes [27]. Bao et al. demonstrated that ECM-receptor interaction, as a key signaling pathway, has been identified as likely to be involved in breast cancer development [28]. Previous similar study by Zhang et al. pointed out that the specific differentially expressed genes in rectal adenocarcinoma were involved in tumor processes, such as proliferation, invasiveness, and metastasis [29], and another research on gastric cancer by Li et al. has proved it as well [30].

In the present study, we further analyzed the interaction mechanism of circRNAs, mRNAs, and miRNAs in BC to examine their correlation with clinical features.

This study showed there were 12 downregulated DEGs and 2 upregulated DEGs in BC samples, as well as 9 interactions. In addition, a total of 5 hub genes including EIF4EBP1, DUSP1, EGR2, EZH1, and CBX7 were correlated with overall survival of BC patients. In brief, EIF4EBP1 was found to be highly expressed, and the remaining four DEGs, including DUSP1, EGR2, EZH1, and CBX7, were displayed in low expression in BC patients. In the research of renal cell carcinoma, Wan et al. suggested that EIF4EBP1 expressions were decreased by the regulation of bromodomain testis-specific protein, with the result of attenuating the increase of tumors [31]. hsa-miR-125b-5p is a miRNA that has already become a biomarker for cancer diagnosis, treatment, and prognosis [32]. We observed that hsa-miR-125b-5p interacted with EIF4EBP1 to modulate the progress of BC. Akbarian et al. also pointed out that EIF4EBP1 was upregulated in multiple sclerosis patients compared to healthy controls [33]. Tumor progression can usually be reflected by DUSP1, which stimulates the progression of tumor after drug resistance. A study confirmed that DUSP1 expression was associated with gefitinib resistance in non-small-cell lung cancer [34], [35]. EGR2 is found to maintain the immune function, promote adaptive immune response, control inflammation, and prevent the development of autoimmune diseases [36]. According to the data we observed, hsa-miR-93-5p was negatively correlated with EGR2 expressions, which was similar to other studies, suggesting that miR-224-5p promotes cell migration, invasion, and epithelial-mesenchymal transition in papillary thyroid carcinoma by targeting EGR2 [37] and indicating that miR-17-5p has a negative regulation to EGR2 in thyroid cancer [38]. EZH1 and CBX7 are genetic regulatory proteins, which are involved in cell proliferation and cancer progression [39]. This study revealed that there was a negative correlation between hsa-miR-93-5p and EZH1, as well as hsa-miR-181b-5p and CBX7. Yamagishi et al. indicated that overexpression of EZH1 and EZH2 was related to the pathogenesis of highly malignant tumors [39]. In addition, Ni et al. indicated that miRNA-21 was found to downregulate CBX7 via the activation of AKT-NF-*κ*B pathway in gastric cancer [40].

The findings in the cancerous and tumor-free breast tissues using RT-qPCR were proved, which confirmed the reliability of our bioinformatics analysis. However, our study still has some limitations. Firstly, the number of samples of normal tissue is not very large. Secondly, the lack of follow-up data about 2 years after operation makes it impossible to conduct a comprehensive survival study. In the future, once we get enough follow-up information, we will verify our analysis results. In conclusion, our study identifies 5 pairs of upcircRNA-downmiRNA-upmRNA network and 20 pairs of downcircRNA-upmiRNA-downmRNA network. The expression level of EIF4EBP1 was increased and the expression levels of DUSP1, EGR2, EZH1, and CBX7 were decreased in cancerous breast tissues compared to tumor-free breast tissues. EIF4EBP1, DUSP1, EGR2, EZH1, and CBX7 were found to be correlated with overall survival of the patients with BC. This study provides a novel perspective to study circRNA-miRNA-mRNA network in BC and assists in the identification of new potential biomarkers to be used for diagnostic and prognostic purposes.

## Figures and Tables

**Figure 1:** Identification of DEmiRNAs, DEmRNAs, and DEcircRNAs between BC and normal breast tissue samples by differentially analyzing the RNA sequencing profile downloaded from TCGA database (1104 BC and 113 normal breast tissue samples) and the GSE101123 dataset (8 BC and 3 normal breast tissue samples) by the volcano plots.

**Figure 2:** DEmRNAs between BC and normal breast tissue samples in BC were analyzed by GO and KEGG pathways. (a) BP, CC, and MF categories (the top 15 GO terms for each category are listed) revealed remarkable enrichment of DEmRNAs. (b) Pathways significantly enriched by the DEmRNAs in the KEGG database; red indicates small *p* value and blue indicates large *p* value; the size of the bubbles indicates the degree of enrichment, and larger bubbles reflect larger gene ratio.

**Figure 3:** Regulatory network of circRNA-miRNA-mRNA in BC was identified. (a) There were 26 pairs of upcircRNA-downmiRNA-upmRNA network. (b) There were 85 pairs of downcircRNA-upmiRNA-downmRNA network.

**Figure 4:** Construction of the PPI network. The interaction of two proteins was reflected by the lines between two nodes; more key location in the PPI network was represented by multiple lines. Upregulated hub genes were revealed in orange color and downregulated hub genes were revealed in green color.

**Figure 5:** Key circRNA-miRNA-mRNA in subnetwork. (a) 5 pairs of key upcircRNA-downmiRNA-upmRNA network. (b) 20 pairs of key downcircRNA-upmiRNA-downmRNA network.

**Figure 6:** Prognostic value of hub-gene signature in BC. A total of 5 hub genes, EIF4EBP1, DUSP1, EGR2, EZH1, and CBX7, were found to be correlated with overall survival of the patients with BC.

**Figure 7:** Expression patterns of EIF4EBP1, DUSP1, EGR2, EZH1, and CBX7 in BC using the starBase database.

**Figure 8:** Expression levels of EIF4EBP1, DUSP1, EGR2, EZH1, and CBX7 in the cancerous (*n* = 48) and tumor-free breast tissues (*n* = 48) by RT-qPCR analysis. *∗* represents *p* < 0.0001 compared with tumor-free breast tissues.

**Table 1:** Primer sequences used for RT-qPCR analysis.

Target	Primer sequences (5′-3′)
EIF4EBP1	F: 5′-TGCGCAATAGCCCAGAAGAT-3′
	R: 5′-TGAGCTGCTCCTTAGAGGGT-3′

DUSP1	F: 5′-TCGCTGCGAAGGACATTTGGG-3′
	R: 5′-AGCGACGCTTCCTGTAAACCC-3′

EGR2	F: 5′-GTCCCCTCGCCGAGCTATTA-3′
	R: 5′-CCGAGCCCGTGTATGCAAAT-3′

EZH1	F: 5′-ACCTTTGCACCCATATTTGCC-3′
	R: 5′-GAGGAATGCTTTATTTCCAGGC-3′

CBX7	F: 5′-GTCAGAGCCATCGCTTCTACT-3′
	R: 5′-ACCTTACCAGGACAGGGTGA-3′

GAPDH	F: 5′-ATGGAGAAGGCTGGGGCTC-3′
	R: 5′-AAGTTGTCATGGATGACCTTG-3′

**Table 2:** Key circRNA-miRNA-mRNA in subnetwork.

	CircRNA	miRNA	mRNA
UpcircRNA-downmiRNA-upmRNA	hsa_circ_0000069	hsa-miR-125b-5p	EIF4EBP1
	hsa_circ_0000512	hsa-miR-296-5p	HMGA1
	hsa_circ_0000513	hsa-miR-296-5p	HMGA1
	hsa_circ_0000514	hsa-miR-296-5p	HMGA1
	hsa_circ_0000515	hsa-miR-296-5p	HMGA1

DowncircRNA-upmiRNA-downmRNA	hsa_circ_0000376	hsa-miR-106b-5p	EZH1
	hsa_circ_0000376	hsa-miR-106b-5p	RRAGD
	hsa_circ_0000376	hsa-miR-106b-5p	CRY2
	hsa_circ_0000376	hsa-miR-181b-5p	CBX7
	hsa_circ_0000376	hsa-miR-200b-3p	JUN
	hsa_circ_0000376	hsa-miR-200b-3p	KDR
	hsa_circ_0000376	hsa-miR-200b-3p	WASF3
	hsa_circ_0000376	hsa-miR-200c-3p	DUSP1
	hsa_circ_0000376	hsa-miR-200c-3p	KDR
	hsa_circ_0000376	hsa-miR-32-5p	PER2
	hsa_circ_0000376	hsa-miR-32-5p	KAT2B
	hsa_circ_0000376	hsa-miR-32-5p	TEF
	hsa_circ_0000376	hsa-miR-429	WASF3
	hsa_circ_0000376	hsa-miR-92b-3p	TEF
	hsa_circ_0000376	hsa-miR-92b-3p	KAT2B
	hsa_circ_0000376	hsa-miR-92b-3p	PER2
	hsa_circ_0000376	hsa-miR-93-5p	CRY2
	hsa_circ_0000376	hsa-miR-93-5p	RRAGD
	hsa_circ_0000376	hsa-miR-93-5p	EGR2
	hsa_circ_0000376	hsa-miR-93-5p	EZH1

## Data Availability

The RNA sequencing profile and the GSE101123 dataset supporting the results displayed in the study could be downloaded from TCGA database (https://tcga-data.nci.nih.gov/) and the GEO database (https://www.ncbi.nlm.nih.gov/gds), respectively.
